RETRACTED

# Green synthesis of Ag/Fe_3_O_4_ nanoparticles using *Mentha longifolia* flower extract: evaluation of its antioxidant and anti-lung cancer effects

**DOI:** 10.1016/j.heliyon.2022.e12326

**Published:** 2022-12-10

**Authors:** Lei Wang, Bikash Karmakar, Fatimah A. Al-Saeed, Ali A. ٍShati, Mutasem Z. Bani-Fwaz, Attalla F. El-kott

**Affiliations:** a Department of Respiratory and Critical Care Medicine, Tianjin Chest Hospital, Tianjin City, 300222, China; b Department of Chemistry, Gobardanga Hindu College, 24 Parganas (North), India; c Department of Biology, College of Science, King Khalid University, Abha, 61421, Saudi Arabia; d ‏Research Center for Advanced Materials Science (RCAMS), King Khalid University, P.O. Box 9004, Abha, 61413, Saudi Arabia; e Department of Chemistry, College of Science, King Khalid University, P. O. Box 9004, Abha, 61413, Saudi Arabia; f Department of Zoology, Faculty of Science, Damanhour University, Damanhour, 22511, Egypt

**Keywords:** Ag nanoparticles, Magnetic nanocomposite, Green synthesis, Lug cancer

## Abstract

Herein, a bio-inspired synthetic method for Ag NP adorned biofunctionalized magnetic nanocomposite has been demonstrated. In the procedure, *Mentha longifolia* flower extract was employed as a template for the green reduction of immobilized Ag ions to corresponding NPs and subsequent stabilization. The phytochemical modification also facilitated the Fe_3_O_4_ NPs to protect from self-aggregation. The as-synthesized Ag/Fe_3_O_4_ nanocomposite material was characterized by SEM, TEM, EDX, elemental mapping, VSM, XRD and ICP-OES methods. Towards the biological application, the material was first explored in the anti-oxidant study following DPPH assay and it exhibited a significant radical scavenging capacity. The application of Ag/Fe_3_O_4_ nanocomposite was further progressed in the anticancer study against standard human lung cancer cell lines (A549 and H358). Cytotoxicity of the material against the cell lines were determined in terms of % cell viability following MTT method and was found to decrease with increase in the material load.

## 1 Introduction

In scientific research and development the concept of nanotechnology has been a ubiquitous phrase these days. It deals with the study and application of nanodimensional materials, usually within the range of 100 nm [1, 2]. Nanometric size of the particles afford large surface to volume ratio and large number of surface active atoms that in turn generates several unique optical, electronic, catalytic and biological properties, being quite different from their macro and micro-counterparts [3, 4]. Their sizes can be tuned into different scales and of diverse shapes like spherical, triangular, rod-like, tubular, star and polyhedral by varying the different reaction conditions like solvent, temperature, pressure, time of reaction, nature of reducing agents etc. [5, 6]. Based on their shape and site selective properties these featured NPs have been used in various domains such as biosensors, electrochemical sensors, wastewater treatment, forensic investigation, hologram printing, catalysis, and biomedical applications [7, 8, 9, 10, 11, 12].

RETRACTED

Despite the presence of several efficient physical, chemical and biological procedures for the synthesis of noble metal NPs, many of them involved unsafe and harmful chemicals as reducing agents, high energy and high pressure procedures for NPs crystallizations, use of carcinogenic solvents, expensive reagents and hazardous methods, which overall made the procedure non-sustainable [13]. Nevertheless, the green and bio-inspired procedures concerning microorganisms (virus, bacteria, fungi, algae), biomolecules (carbohydrates, lipid, proteins, polymers) and plant extracts are much safer, non-toxic, inexpensive and also the corresponding materials are biodegradable and biocompatible [14, 15, 16, 17, 18, 19, 20, 21, 22]. Now, among these protocols, the plant based biosynthesis of NPs has been more advantageous as, i) it is absolutely green and energy efficient involving water as reaction media at ambient conditions, ii) no chance of microbial contamination which is mandatory in biological applications, iii) *in situ* green reduction of metal ions into NPs facilitated by the phytomolecules of plant, averting harsh reducing agents, iv) providing additional stabilization to NPs by biomolecular encapsulation and v) non-aggregated uniform sized particles [23, 24, 25, 26, 27, 28]. Being inspired, several research articles have been published on plant (leaves, flower, fruit, seed, root, bark, gum etc) extract mediated biogenic synthesis [29, 30, 31]. Following the trend [32], we herein demonstrate the architecture and synthesis of *Mentha longifolia* or mint flower extract templated sustainable synthesis of Ag NPs impregnated magnetic Fe_3_O_4_ NPs, as a magentically retrievable bio-nanocomposite material. *Mentha* is a perennial herb that grows abundantly in the moist atmosphere. It is rich in phytochemicals like monoterpenes and monoterpenoids (menthol, menthone, isomethone, neomethol, piperitone, α/β-pinene), sesquiterpene (β-caryophyllene), different kinds of tannins and flavonoids [33, 34]. Mostly these are oxygenated compounds and the electron rich organofunctions facilitate the *in situ* green reduction of Ag ions. Since these tiny Ag NPs have high affinity to self-aggregate, we allowed them to disperse over pre-synthesized Fe_3_O_4_ NPs. The as-synthesized nanocomposite seem also advantageous in terms of easy magnetic isolation from the system [35].

RETRACTED

Some recent literatures have revealed the significant cancer diagnosis and therapeutic potential of bio-engineered noble metal NPs like Cu, Au and Ag NPs [36, 37]. It's pretty wondering to see the superior use and application of bio-functionalized NPs over conventional cancer therapy. Some important reasons behind that is the toxicity and side effects produced by them due to non-specific targeting in the body cells, drug-resistance on the body, quick drug metabolism and clearance from the patient's body, expensiveness of the treatment procedure etc [13]. Mechanistically, different biofunctionalized nanoformulated noble metal composites easily enter the cancer cells through endocytosis and surpass the blood-brain barrier (BBB) due to their compatible sizes and environment. They spread all over the cytoplasm and nucleus by intracellular trafficking, damage the mitochondrial function and generates reactive oxygen species (ROS) around their surface. Subsequently, they enhance the secretion of lactate dehydrogenase enzyme to deregulate the cell cycle and finally lead to apoptosis. Ag NPs have been found very efficient in generating ROS in the cell environment and also exhibit significant antiangiogenicand anti-proliferative properties [38, 39, 40, 41, 42, 43, 44, 45, 46].

Being encouraged by these, we are prompted to employ the novel Ag/Fe_3_O_4_ nanocomposite material towards inhibiting the growth of human lung cancer. In addition we also studied its antioxidant potential which is believed to be related with the anticancer activity (see Scheme 1).

**Scheme 1:** Schematic green synthesis of Ag/Fe_3_O_4_ nanocomposite mediated by *Mentha longifolia* flower extract.

## 2 Experimental

### 2.1 Preparation of *Mentha longifolia* flower extract

1.0 g of dried *Mentha longifolia* flower were washed thoroughly with double distilled water and extracted in 50 mL DI water by boiling at 60 °C for 20 min. It was filtered through Whatman-1 filter paper and the pale yellow colored filtrate was used as the mentha extract.

### 2.2 Green synthesis of the Ag/Fe_3_O_4_ nanocomposite

Fe_3_O_4_ NPs were pre-synthesized following recent literature. 0.5 g of material was dispersed in deionized water (50 mL) by sonication for 30 min. The precursor of Ag ions, AgNO_3_, was added to the mixture (0.03 g) under stirring and continued for 30 min for immobilization of Ag ions over Fe_3_O_4_. Subsequently, *Mentha longifolia* flower extract was introduced to initiate the green reduction. The mixture was stirred for another 60 min and the Ag/Fe_3_O_4_nanocomposite formed was isolated magnetically, washed with deionized water and dried at 60 °C.

RETRACTED

### 2.3 Investigation of antioxidant activity

In the study of antioxidant activity of Ag/Fe_3_O_4_ nanocomposite, the DPPH (1,1-diphenyl-2-picrylhydrazil) radical scavenging assay was followed. A methanolic solution of DPPH radical was brought in contact to the experimental antioxidant material in different concentration when the radical gets quenched by abstracting protons or free electrons it. This makes a visible change in color from violet to pale yellow. The antioxidant capacity is determined in terms of % inhibition by spectroscopic measurement following Eq. (1).

(1) $$Inhibition\left(\%\right)=\left(1-\frac{Abs_{sample}-Abs_{blank}}{Abs_{control}-Abs_{blank}}\right)\times 100$$

*Abs sample:* absorbance of the reaction mixture, *Abs blank:* absorbance of the blank for each sample dilution in DPPH solvent, *Abs control*: absorbance of DPPH solution in sample solvent.

### 2.4 Investigation of cytotoxic activity

The cell lines were initially cultured in 96-well plates at 37 °C in 5% CO_2_ atmosphere for 24 h. The growth media (10% FBS) was then decanted off from the plate and were washed twice with PBS. The compounds were then introduced in different concentrations (0.5, 5, 50, 500, and 1000 μg/mL) in RPMI medium and the system was incubated again for 3 days. The MTT dye in PBS solution (10 μL, 5 mg/mL) was next added to each well and incubated again for 4 h. In the same way media was removed and replaced with 100μL DMSO in each well. In order to assist the formazan crystal solubilization all the plates were gently swirled. Finally, absorbance of the resulting mixture was measured at 545 nm and % cell toxicity alongwith IC 50 were determined as following Eq. (2).

(2) $$\text{T}\text{o}\text{x}\text{i}\text{c}\text{i}\text{t}\text{y}\;\%=\left(1-\frac{\text{m}\text{e}\text{a}\text{n}\;\text{OD}\;\text{of}\;\text{sample}}{\text{m}\text{e}\text{a}\text{n}\;\text{OD}\;\text{of}\;\text{control}}\right)\times 100$$

Viability%=100−Toxicity%

## 3 Results and discussion

### 3.1 Characterization and data analysis of Ag/Fe_3_O_4_ nanocomposite

The Ag/Fe_3_O_4_nanocompositewas prepared following a stepwise modification approach. This involves the initial synthesis of Fe_3_O_4_ NPs by co-precipitation method followed by the impregnation of Ag ions over them. The composite as formed was then biogenically reduced over *Mentha longifolia* flower extract to produce the final material.

After the synthesis, the nanocomposite material definitely demands its physical characterizations, which was carried out over SEM, TEM, EDX, elemental mapping, XRD and VSM analysis. At the outset we studied the surface texture, particle shape and dimension, and their relative dispersion. Figure 1 clearly displays the two different kind of NPs, one for extract modified Fe_3_O_4_ (Figure 1a) and another for hybrid Ag/Fe_3_O_4_ nanocomposite (Figure 1b) having grey and black color respectively. Both the kind are almost globular in shape. Evidently, the Ag NPs are of larger size (35–40 nm) than Fe_3_O_4_ NPs (10–15 nm). It looks as the two kinds of particles are encapsulated inside a gel like appearance, which is undoubtedly the *Mentha longifolia* flower extract biomolecular coating. Due to this kind of arrangement the particles are quite apart from each other and free from aggregation. The SEM image of Ag/Fe_3_O_4_ nanocomposite, as shown in Figure 2, also verifies the spherical shaped nanocomposite particles. Although, their individual recognition could not be done from the SEM investigation. It is due to manual sampling the material looks agglomerated.

RETRACTED

**Figure 1:** TEM images of (a) Fe_3_O_4_/extract NPs and (b) Ag/Fe_3_O_4_ nanocomposite.

**Figure 2:** SEM image of Ag/Fe_3_O_4_ nanocomposite.

Next we had the elemental composition study, which was done through EDX analysis, being equipped with the SEM instrument. Figure 3 clearly demonstrates the corresponding profile of Ag/Fe_3_O_4_ nanocomposite with the presence of Fe and Ag as metallic component and C and O as non-metals. A major broad signal of Au is observed at 2.1 keV, which is attributed to the Au vapor deposition over the nano-sample prior to analysis, and not of the sample component. The non-metals obviously account for the *Mentha longifolia* flower extract phytomolecular association with the sample matrix. We further validated the EDX results and concreted the information with elemental mapping study. This offers an excellent comprehension of atomic dispersion of the constituent elements over the surface. As Figure 4 depicts, X-ray scanning of a section of the SEM image generates the signals in the form of dots which represent the corresponding elemental species. Markedly, they are homogenously distributed over the surface which has a significant impact in showing superior activity.

**Figure 3:** EDX spectrum of Ag/Fe_3_O_4_ nanocomposite.

**Figure 4:** SEM image of Ag/Fe_3_O_4_ nanocomposite with its elemental mapping.

The crystallinity and nature of diffraction phases of Ag/Fe_3_O_4_ nanocomposite was determined by XRD analysis, which has been shown in Figure 5. Fe_3_O_4_ NPs can be recognized from its nature of diffractions on (220), (311), (400), (422), (511) and (440) Fe_3_O_4_ crystal planes which appeared on 2θ angles of 31.3, 36.4, 44.2, 54.8, 58.4 and 64.3°. These angles resemble closely with the standard JCPDS values (File No 19-0629). In addition, some weak diffraction peaks related to Ag NPs are observed at 2θ = 41.2°, 45.1°, 62.3° and 77.4°, attributed to *fcc* silver (111), (200), (220) and (311) crystal planes. The broad and non-crystalline region in the 10-15° angles corresponds to the *Mentha longifolia* flower extract phytochemicals. Calculating the FWHM (Full Width at Half Maxima) values, Scherrer's formula (D = Kλ/βcosθ) has been used to determine the particle size of the Ag/Fe_3_O_4_ nanocomposite, which appeared to be 48.4°. However, the same for un-doped Fe_3_O_4_ was found as 17.3°. This is fairly close to the dimension predicted from TEM analysis.

RETRACTED

**Figure 5:** XRD pattern of Ag/Fe_3_O_4_ nanocomposite.

As the material contained Fe_3_O_4_ at its core, the study of its magnetic properties was felt very important and accordingly VSM analysis was carried out. Exposing the Ag/Fe_3_O_4_ nanocomposite to a variable magnetic field within the range of -20 kOe to +20 kOe produces the resultant profile in the form of a magnetic hysteresis curve, being shown in Figure 6. This justifies the material to be of paramagnetic nature. The related magnetization saturation (Ms) value obtained as 40.5 emu/g. This value is however much less from the unmodified pristine Fe_3_O_4_ NPs. The doping of non-magnetic Ag NPs as well as flower extract phytochemicals are responsible for the decrease in magnetism significant. However, it was sufficiently magnetic to be retrieved by external magnet.

**Figure 6:** VSM analysis of Ag/Fe_3_O_4_ nanocomposite.

### 3.2 Antioxidant activity of Ag/Fe_3_O_4_ nanocomposite

The Ag/Fe_3_O_4_ nanocomposite material was first subjected to the study of antioxidant competence. In earlier studies it has been reported that a material having significant antioxidant capacity, exhibits very good resistance to proliferation of cancer and apoptosis of the malignant cells. The well known DPPH radical scavenging investigation was carried out in this regard and the corresponding result is represented in Figure 7. As it shows, the Ag/Fe_3_O_4_ nanomaterial was used in diverse concentrations, i.e., 31.25, 62.5, 125, 250, 500 and 1000 μg/mL to react with the DPPH methanol solution and the radical quenching potential was increased gradually with material concentration. Mechanistically, the material under investigation transfers an electron or hydrogen to the DPPH free radical and reduces it to a stable molecular species. This change is manifested by a visible color change from purple to pale yellow. Spectrophotometric (UV-Vis spectroscopy) measure of this process is carried out at a wavelength of 517 nm and the antioxidant properties were finally calculated following Eq. (1). Markedly, the radical scavenging capacity of Ag/Fe_3_O_4_ nanomaterial was enhanced with increasing concentrations and became highest (92%) at 1000 μg/mL (Figure 7).

RETRACTED

**Figure 7:** Antioxidant activity of Ag/Fe_3_O_4_ nanocomposite.

### 3.3 Cytotoxicity studies over Ag/Fe_3_O_4_ nanocomposite

On having a significant IC_50_ value in radical scavenging assay for antioxidant investigation, we extended the bio-application of the desired nanocomposite in anticancer study over A549 and H358 human lung cancer cell lines with *in vitro* conditions following the standard MTT assay. The related outcome has been shown in Figures 8 and 9. Interestingly, the % cell viability values over the malignant cell lines reduced dose-dependently in presence of Ag/Fe_3_O_4_ nanocomposite. IC_50_ values of the nanocomposite were observed to be 162.86 μg/mL and 412.23 against the A549 and H358 cell lines respectively. These results evidently suggest the Ag/Fe_3_O_4_ nanocomposite as a novel chemotherapeutic material against the lung cancer cell lines.

**Figure 8:** In *vitro* toxicity analysis of Ag/Fe_3_O_4_ nanocomposite on A549 cell line.

**Figure 9:** In *vitro* toxicity analysis of Ag/Fe_3_O_4_ nanocomposite on H358 cell line.

## 4 Conclusion

To summarize, an eco-friendly and biogenic method for the nano-architechtonic synthesis of Ag/Fe_3_O_4_ composite has been demonstrated using *Mentha longifolia* flower (mint) extract. The electron rich oxygenated phytochemicals acted as a green and natural reducing and as well as stabilization agent. The layering of these biomolecules over Fe_3_O_4_ also prevent them from agglomeration. The as-synthesized material was analyzed by a range of analytical techniques. From TEM analysis, the Ag NPs over the nanocomposite was observed to be almost spherical shaped and uniformly distributed over the support. The two different kind of particles in terms of size and color, attributed to Ag and Fe_3_O_4_ NPs are very clear from the image. XRD analysis afforded the material of high crystallinity. After detailed characterizations, the Ag/Fe_3_O_4_ nanocomposite was explored biologically in the investigation of antioxidant capacity by DPPH radical scavenging assay. After attaining an excellent potential the material was subjected to cytotoxicity and human anti-lung cancer studies against A549 and H358 cell lines. The MTT method was used in determining cytotoxicity in terms of % cell viability or toxicity. The material exhibited gradual increase in % toxicity with increase in its dose. The consequent IC_50_ values were found as 162.86 and 412.23 μg/mL respectively. Hence, the promising potential as shown by the Ag/Fe_3_O_4_ hybrid material in-vitro studies, definitely would project it as a prospective nano-chemotherapeutic drug in near future.

RETRACTED

## Declarations

### Author contribution statement

Lei Wang, Attalla F. El-kott: Conceived and designed the experiments.

Bikash Karmakar: Analyzed and interpreted the data; Wrote the paper.

Fatimah A. Al-Saeed, Mutasem Z. Bani-Fwaz: Performed the experiments.

Ali A. Shati: Contributed reagents, materials, analysis tools or data.

### Funding statement

This work was supported by Tianjin Key Medical Discipline (Specialty) Construction Project (Number: TKYXZDXK-049A) and the Deanship of Scientific Research at King Khalid University.

### Data availability statement

Data will be made available on request.

### Declaration of interests statement

The authors declare no conflict of interest.

### Additional information

No additional information is available for this paper.
